The article "The Clinical Efficacy and Safety of Extracorporeal Shock Wave Lithotripsy in the Treatment of Patients with Urinary Calculi" was retracted in 2023. Reasons: unreliable results or conclusions; lack of ethics approval or compliance; concerns about the data; concerns about the peer review.

# The Clinical Efficacy and Safety of Extracorporeal Shock Wave Lithotripsy in the Treatment of Patients with Urinary Calculi

**DOI:** 10.1155/2022/3468692

**Published:** 2022-10-13

**Authors:** Dazhao Zhang, Zhiheng Liang, Daming Wang, Jie Lv, Demao Ding, Dexin Yu

**Affiliations:** ^1^Department of Urology, The Second Affiliated Hospital of Anhui Medical University, Hefei 230032, China; ^2^Department of Urology, Sinopharm Dongfeng General Hospital, China

## Abstract

**Objective:**

To evaluate the clinical efficacy of extracorporeal shock wave lithotripsy (ESWL) for urinary calculi and precautions of postoperative complications.

**Methods:**

90 patients with urinary calculi at our hospital were randomly recruited between July 2019 and July 2020 and were allocated (1 : 1) to receive either ESWL (observation group) or conventional surgery (control group). Clinical efficacy was the primary endpoint, whereas adverse events were the secondary endpoint.

**Results:**

The operation time, early activity time, and hospitalization time of the observation group were significantly lower than those of the control group (*P* < 0.05). ESWL resulted in less postoperative pain in patients versus conventional surgery (*P* < 0.05). ESWL was associated with a significantly higher total clinical efficacy (97.78%) versus conventional surgery (82.22%) (*P* < 0.05). The eligible patients given ESWL had a lower incidence of complications (11.12%) versus those given conventional surgery (31.12%) (*P* < 0.05).

**Conclusion:**

Hematuria prevention requires precise localization of stones as well as adjustment of pulse energy and the number of impacts due to stone changes. Precautions against renal colic necessitate complete comminution of stones intraoperatively, more postoperative water intake, moderate exercise, or injection of antispasmodic drugs and cathartics for pain relief. Nausea and vomiting precautions require preoperative recording of previous medical history and corresponding treatment, intraoperative real-time adjustment of voltage pulse frequency, and duration depending on the magnitude of intraoperative reaction. Urinary tract infection prevention requires preoperative prevention and proper postoperative anti-infection and anti-inflammatory treatment, along with enough water intake and bed rest. Other precautions include thorough comminution of the calculi, proper anti-infection and anti-inflammatory treatment, no early exercise or excessive activity after surgery, and proper postoperative care. ESWL is effective in treating patients with urinary calculi with a simple, safe, and quick operation and a low incidence of adverse events, as it effectively reduces the incidence of complications, accelerates the recovery of patients and improves their quality of life.

The article "The Clinical Efficacy and Safety of Extracorporeal Shock Wave Lithotripsy in the Treatment of Patients with Urinary Calculi" was retracted in 2023. Reasons: unreliable results or conclusions; lack of ethics approval or compliance; concerns about the data; concerns about the peer review.

## 1. Introduction

Urinary calculi are a common disease [1] with clinical manifestations such as abdominal distension, nausea, vomiting, hematuria, colic, and, in severe cases, hydronephrosis and renal function impairment [2, 3]. Patients with urinary calculi are mostly aged 25-40 years [4], and only 2-3% of cases are found in children aged 2-6 years, which is frequently associated with urinary tract infections and congenital malformations [5]. Urinary calculi can be found in any part of the kidney, bladder, ureter, and urethra, with kidney and ureteral stones being the most common. Type 2 diabetes is a systemic metabolic disease caused by insufficient insulin secretion or resistance in the body. It is a common and frequently occurring disease among middle-aged and elderly people, which not only affects the blood glucose metabolism in the body but also is related to the occurrence of multiple diseases in multiple systems of the body, such as circulation, urinary tract, and blood coagulation. Urinary calculi are not uncommon in clinical practice, and it is currently believed that there is a certain correlation between them and diabetes. The formation of urinary calculi may be related to two major factors, infection and metabolism. Therefore, metabolic syndromes such as T2DM, hypertension, hyperlipidemia, and obesity may be related to the formation of calculi.

Currently, the incidence of urinary stones in China is 1%-5% [6], 25% of which require hospitalization. Diabetes, according to studies, increases the recurrence incidence of urinary calculi following therapy by 2 to 3.5 times that of nondiabetic calculi patients. Repeated stone formation is linked to a cascade of metabolic kidney damage (such as oxalic acid, cystine, and uric acid-related nephropathy), culminating in patients' impaired renal function [7]. More seriously, patients with urinary calculi combined with diabetes are prone to complications after surgery, such as urinary tract obstruction, and infection, further aggravating the damage of renal function, leading to end-stage renal disease, and eventually facing dialysis or kidney transplantation. Diabetic patients have low immunity and are vulnerable to various infections, among which urinary tract infection is the most common [8].

The current conservative treatment regarding urinary stones includes the consumption of water, exercise, and anti-inflammation. Urinary calculi belong to the category of “stone stranguria” in traditional Chinese medicine, which is one of the five stranguria, and its treatment principle should be clearing away heat and dampness, expelling stone and dredging stranguria. TCM formulas for urinary stones include (1) granules, such as Paishi Granules, Hupo Xiaoshi Granules, Fufang Jinqiancao Granules; (2) tablets, such as Xiaoshi tablets, Jieshitong Tablets, and Shilintong tablets; (3) capsules, such as Jingshiling capsules and Mishitong capsules; and (4) other dosage forms, such as Niaoshitong pills and Shenshitong powder. Due to the ineffectiveness of drug treatment, surgery is currently the mainstay of treatment [9]. Traditionally, ureteral stones are treated mainly by surgical excision and pneumatic bomb lithotripsy. With the continuous improvement of modern urolithiasis treatment technology, many new treatment techniques such as ultrasound lithotripsy and holmium laser lithotripsy have been gradually developed. Ultrasound lithotripsy is available for patients with mild urinary stones, and common procedures in the surgical treatment of severe urinary stones include pneumatic ballistic lithotripsy and holmium laser lithotripsy, which effectively improves the effective removal rate of the procedure through ureteroscopic guidance. Conventional urinary calculi treatment mostly adopts surgical stone extraction, but it is highly traumatic with great difficulty in thorough stone removal and fails to reduce the high recurrence rate.

The article "The Clinical Efficacy and Safety of Extracorporeal Shock Wave Lithotripsy in the Treatment of Patients with Urinary Calculi" was retracted in 2023. Reasons: unreliable results or conclusions; lack of ethics approval or compliance; concerns about the data; concerns about the peer review.

Thus, there exists an urgent need to explore appropriate treatment methods for pain relief, obstruction elimination, and renal function protection. Extracorporeal shock wave lithotripsy (ESWL) [10] is one of the minimally invasive treatments of upper urinary tract stones with well-recognized efficacy [11]. ESWL is a noninvasive approach for treating stones using an extracorporeal lithotripter to target and emit shock waves repeatedly to break up the stones and allow their evacuation from urine [12]. However, there are concerns about the complications associated with high-energy shock waves [13]. Accordingly, this study was conducted to evaluate the clinical efficacy of ESWL for urinary calculi and precautions for postoperative complications.

## 2. Materials and Methods

### 2.1. Baseline Data

Between July 2019 and July 2020, 90 patients with urinary calculi in our institution assessed for eligibility were randomly recruited. They were concurrently assigned to either an observation group (*n* = 45) or a control group (*n* = 45).

The randomization was carried out using an online web-based randomization tool (freely available at http://www.randomizer.org/). For concealment of allocation, the randomization procedure and assignment were managed by an independent research assistant who was not involved in the screening or evaluation of the participants.

The article "The Clinical Efficacy and Safety of Extracorporeal Shock Wave Lithotripsy in the Treatment of Patients with Urinary Calculi" was retracted in 2023. Reasons: unreliable results or conclusions; lack of ethics approval or compliance; concerns about the data; concerns about the peer review.

We estimated that with a sample size of 45 patients assigned to receive ESWL and 45 assigned to receive conventional surgery, the study would have more than 99% power to detect a between-group difference in the relevant indicators for this study.

The study protocol and all amendments were approved by the appropriate ethics committee at each centre. The study was done in accordance with the protocol, its amendments, and standards of Good Clinical Practice. All participants provided written informed consent before enrolment (ethics number: MI-YU20190706).

The baseline characteristics of the patients in the observation group were comparable with those of the control group (*P* > 0.05) (Table 1).

### 2.2. Inclusion and Exclusion Criteria

Inclusion criteria are as follows: ① patients were diagnosed with urinary stones by ultrasound, X-ray, or intravenous urography, ② patients were informed about the study and provided informed consent, ③ in line with the surgical indications, and ④ with complete clinical data.

Exclusion criteria are as follows: ① patients with contraindications to relevant treatment; ② with renal insufficiency, abnormal cardiopulmonary function, or abnormal coagulation function; ③ with unconsciousness or psychiatric disorders; ④ with peripheral bleeding disorders; ⑤ with cerebral hemorrhage and hypertension six months before surgery; ⑥ with hepatitis and atypical pneumonia; ⑦ with diabetes mellitus, pregnancy or during menstruation; and ⑧ with renal dysfunction and urinary tract infection.

### 2.3. Methods

The patients in the control group were treated with conventional surgery. The specific operations are as follows: prepare the impact rod and ureteroscope, insert the impact rod into the ureteroscope, and connect the lithotriptor when the stone is pressed against the ureteral wall to crush the stone. After that, the ureteral stone forceps were used to remove the slightly larger calculi after crushing, and the smaller calculi flowed out spontaneously through the ureteral drainage tube.

The observation group were given ESWL using an XT03C extracorporeal shock wave lithotripsy machine. In the case of stones in the pelvic and intramural segments of the ureter and the bladder, the stones were detected in the prone position with the external iliac artery and the common iliac artery on the affected side as markers. In the case of stones in kidney stones, upper and middle ureter, the lesion was observed in a supine position, and the lithotripter probe was adjusted to the position where the stones and the posterior image were clearly visualized, and the stones were observed by double images. To observe another image, the midline of the image screen on one side was frozen at the location of the stone acoustic adjustment site, after which the distance from the stone to the epidermis was measured, followed by observation of the image and positioning. The lithotripter was then activated for lithotripsy, and the voltage was increased according to the energy loss and patient's tolerance, with a common voltage of 7-13 kV, 40-50 shocks per minute, 800-1200 shocks per session, depending on the degree of stone comminution, and a lithotripsy interval of 7-30 d. Patients with multiple stones require anti-infection treatment after lithotripsy and were advised to drink more water and exercise after the procedure to facilitate lithotripsy discharge.

The article "The Clinical Efficacy and Safety of Extracorporeal Shock Wave Lithotripsy in the Treatment of Patients with Urinary Calculi" was retracted in 2023. Reasons: unreliable results or conclusions; lack of ethics approval or compliance; concerns about the data; concerns about the peer review.

### 2.4. Clinical Endpoints

1. Surgical index level: the operation time, early activity time, and hospitalization time of the two groups of patients were recorded
2. Pain score: the visual analogue scale (VAS) was used for evaluation. The total score was 10 points. The score was proportional to the severity of pain. Zero points represented no pain, 10 points represented the most severe pain, and 0-3 points means mild pain, which is tolerated and does not affect daily life; 4-6 points means moderate pain, which requires adjuvant treatment with analgesics; 7-10 points means severe pain, intolerable, and seriously affecting sleep
3. Urinary red blood cell number and stone expulsion time: the number of urinary red blood cells and the stone excretion time were recorded
4. Stone removal: the one-time success rate of lithotripsy and the stone removal rate were recorded in detail, and the stone removal status of the two groups of patients was compared
5. Clinical efficacy: clinical efficacy is divided into markedly effective, effective, and ineffective. Markedly effective: the stones were completely removed, the symptoms of hematuria and lumbar pain disappeared completely, and there were no residual stones after X-ray and ultrasound examination. Effective: symptoms such as hematuria and lumbar pain were alleviated, and patients had residual stones by X-ray and ultrasound examination. Ineffective: no significant difference was found in the comparison between before and after treatment. Total efficacy = (markedly effective + effective)/total number of cases × 100%
6. Complications: postoperative complications included hematuria, renal colic, nausea and vomiting, urinary tract infection, and lithotripsy accumulation. The incidence of complications was calculated, and their causes and preventive measures were analyzed

### 2.5. Statistical Analysis

If the parameter beta is either a difference of means, a log odds ratio, or a log hazard ratio, then it is reasonable to assume that b is unbiased and normally distributed.

The article "The Clinical Efficacy and Safety of Extracorporeal Shock Wave Lithotripsy in the Treatment of Patients with Urinary Calculi" was retracted in 2023. Reasons: unreliable results or conclusions; lack of ethics approval or compliance; concerns about the data; concerns about the peer review.

SPSS 22.0 was used for data analyses. The measurement data were expressed as ($\bar{x}\pm s$) and processed using the *t*-test. The count data were expressed as the number of cases (rate) and analyzed using the chi-square test. Differences were considered statistically significant at *P* < 0.05.

## 3. Results

### 3.1. Surgical Index Level

The observation group's surgery time, early activity time, and hospitalization time were considerably shorter than those of the control group (*P* < 0.05) (Table 2).

### 3.2. VAS Score

In the control group, there were 28 (62.22%) cases of mild pain, 12 (26.67%) cases of moderate pain, and 5 (11.11%) cases of severe pain. There were 40 (88.89%) cases of mild pain, 5 (11.11%) cases of moderate pain, and 0 (0.00%) cases of severe pain. ESWL resulted in less postoperative pain in patients versus conventional surgery (*P* < 0.05) (Table 3).

### 3.3. The Number of Red Blood Cells in Urine

The amount of urine red blood cells did not differ significantly between the two groups (40.78 ± 8.78, 41.75 ± 9.08) (*P* > 0.05) (Table 4).

### 3.4. Stone Expulsion Time

The stone expulsion time in the control group was significantly shorter than that in the observation group (*P* < 0.05) (Table 5).

### 3.5. Stone Removal

In the control group, there were 32 (71.11%) cases with successful one-time lithotripsy, and 40 (88.89%) cases with stone clearance rate, while those (43(95.56%), 44 (97.78%)) in the observation group was lower (*P* < 0.05) (Table 6).

### 3.6. Clinical Efficacy

There were 21 (46.67%) cases of markedly effective, 23 (51.12%) cases of effective, and 1 (2.22%) case of ineffective in the observation group, and there were 15 (33.34%) cases of markedly effective, 22 (48.89%) cases of effective, and 8 (17.78%) cases of ineffective in the control group. ESWL resulted in a significant higher total clinical efficacy (97.78%) versus conventional surgery (82.22%) (*P* < 0.05) (Table 7).

### 3.7. Complications

There were 2 (4.45%) cases of hematuria, 1 (2.23%) case of renal colic, 1 (2.23%) case of nausea and vomiting, and 1 (2.23%) case of other in the observation group, and there were 6 (13.34%) cases of hematuria, 3 (6.67%) cases of renal colic, 2 (4.45%) cases of nausea and vomiting, 2 (4.45%) cases of urinary tract infection, and 1 (2.23%) case of other in the control group.

The eligible patients given ESWL had a lower incidence of complications (11.12%) versus those given conventional surgery (31.12%) (*P* < 0.05) (Table 8).

#### 3.7.1. Causes

ESWL is a noninvasive method for the treatment of stones using an extracorporeal lithotripter to aim and release shock waves repeatedly to break up the stones and allow their removal from urine. However, improper energy and the number of shocks may cause damage and subsequent complications, and hypertension and diabetes mellitus are important clinical risk factors. The effectiveness of ESWL lithotripsy and the degree of tissue damage is positively correlated with the energy of the pulse beam, and the severity of damage to target tissues by various types of extracorporeal lithotripters is proportional to the number of impacts, so high energy and multiple impacts are the main technical parameters of pathogenesis. Therefore, the use of ESWL should be carried out in strict accordance with the operating procedures, understanding the indications and contraindications, the control of the voltage frequency, and the number of shocks, which could effectively reduce the incidence of complications [14].

The article "The Clinical Efficacy and Safety of Extracorporeal Shock Wave Lithotripsy in the Treatment of Patients with Urinary Calculi" was retracted in 2023. Reasons: unreliable results or conclusions; lack of ethics approval or compliance; concerns about the data; concerns about the peer review.

#### 3.7.2. Precautions

1. Hematuria: it is attributed to damage to the mucosa of the urinary tract elicited by excessive pulse energy and frequent or inaccurate focus during lithotripsy. However, most of the symptoms are mild and will disappear without treatment in 1-2 d. Hematuria prevention requires precise localization of stones and adjustment of pulse energy and the number of impacts according to stone changes
2. Kidney colic: this is caused by incomplete and insufficient stone comminution, resulting in the discharge of the stone into the ureter and pain caused by the ureteral spasm. Precautions against renal colic require complete comminution of stones intraoperatively, more postoperative water intake, moderate exercise, or injection of antispasmodic drugs and cathartics for pain relief
3. Nausea and vomiting: this is triggered by the application of intraoperative pain medication or the frictional stimulation of the ureter during the discharge of the debris or the vagal reflex caused by the stimulation of the pleura by the shock wave. The symptoms are usually mild and will disappear without treatment in 1-2 days. Its precautions require preoperative recording of previous medical history and corresponding treatment, intraoperative real-time adjustment of voltage pulse frequency, and duration depending on the degree of intraoperative reaction
4. Urinary tract infection: it mostly occurs within 6 h after surgery, accompanied by poor stone removal and renal colic, mostly induced by uncontrolled urinary tract infection or blockage of the urinary tract by debris accumulation. Its preventions require preoperative prevention, proper postoperative anti-infection, and anti-inflammatory treatment, along with enough water intake and bed rest
5. Other: other symptoms include steinstrasse and residual stone regrowth. Relevant precautions include thorough comminution of the calculi, proper anti-infection and anti-inflammatory treatment, no early exercise or excessive activity after surgery, and proper postoperative care.

The article "The Clinical Efficacy and Safety of Extracorporeal Shock Wave Lithotripsy in the Treatment of Patients with Urinary Calculi" was retracted in 2023. Reasons: unreliable results or conclusions; lack of ethics approval or compliance; concerns about the data; concerns about the peer review.

## 4. Discussion

The clinical symptoms of urinary stones are abdominal pain and urination disorders. The occurrence of the disease is closely associated with the patient's dietary structure and lifestyle habits, such as excessive intake of high-calcium foods, which increases urinary calcium concentration and forms stones after precipitation [7]. Long-term metabolic abnormalities in the body can lead to blockage of the urinary tract, accelerating crystal aggregation and eventually leading to the occurrence of stones, which severely affects the physical and mental health of patients and compromises their quality of life [15]. Conventional treatment of urinary stones is time-consuming, with residual stone removal and average clinical efficacy. Obstruction of the urethra by stones may inflict lumbar and abdominal cramps, seriously compromising the quality of life of patients. ESWL is associated with accurate localization and comminution of stones [16, 17] and is a noninvasive method that eliminates the trauma of surgery and provides promising therapeutic benefits [18]. Most of the existing studies fail to fully elucidate the mechanisms of formation, and there is no ideal prevention modality for most cases [19].

The results of the present study found that extracorporeal shock wave lithotripsy for the treatment of urinary calculi patients had milder pain after treatment; the number of urinary red blood cells was significantly reduced; the stone expulsion, the operation time, early activity time, and hospitalization time were significantly shortened. Traditional treatment approaches include surgical stone removal; however, this is impracticable due to the risk of intestinal blockage in patients, as well as the high trauma and low patient tolerance. Extracorporeal shock wave lithotripsy focuses shock waves through a lithotripsy equipment to release energy and break up stones. Extracorporeal shock wave lithotripsy fully incorporates the advantages of B-ultrasound and X-ray, realizes the benefits of correct placement, eliminates blind operation, swiftly and thoroughly removes calculi, and has a favorable safety profile in the treatment of urinary calculi. Additionally, extracorporeal shock wave lithotripsy can also reduce tissue adhesion and facilitate the smooth discharge of stones. Extracorporeal shock wave lithotripsy is a minimally invasive procedure that is frequently utilized in clinical therapy owing to its merits of reduced trauma, less kidney damage, and a high lithotripsy rate. This method breaks up the calculi and is especially suited for individuals with ureteral calculi that have been imprisoned for a long period, hard texture, and granulation tissue. Furthermore, with ultrasound guidance, the size, position, and quantity of the stones can be identified prior to treatment, resulting in an increased removal rate of stones. The lumen of the urinary system can be operated during the therapy of transurethral lithotripsy. It effectively avoids the mucosal damage of the urinary system and also shortens the operation time, which is consistent with the previous research results.

The article "The Clinical Efficacy and Safety of Extracorporeal Shock Wave Lithotripsy in the Treatment of Patients with Urinary Calculi" was retracted in 2023. Reasons: unreliable results or conclusions; lack of ethics approval or compliance; concerns about the data; concerns about the peer review.

In the present study, ESWL resulted in a significantly higher total clinical efficacy (97.78%) versus conventional surgery (82.22%) (*P* < 0.05). The basic principle of extracorporeal shock wave lithotripsy is to create a high-temperature, high-pressure plasma zone with a high energy density using a high-voltage, high-current, and instantaneous discharge, which rapidly converts electrical energy into heat, light, force, and sound energy, causing pressure pulses in the aqueous medium and shattering stones under X-ray guidance. In comparison to conventional lithotripsy, ESWL provides lithotripsy efficacy and achieves maximal human protection, with a high safety, dependability, painlessness, and good lithotripsy outcomes [20]. Here, the eligible patients given ESWL had a lower incidence of complication (11.12%) versus those given conventional surgery (31.12%) (*P* < 0.05), indicating that ESWL effectively avoids the defects of conventional surgery with a high safety profile, which is consistent with the results of previous studies. Nonetheless, incorrect ESWL shock wave energy and impact number may cause injury. In general, the intensity of the pulse beam is positively connected with the effectiveness of ESWL lithotripsy and the degree of tissue damage, and the degree of damage to target tissues by various types of extracorporeal lithotripters is proportionate to the number of hits.

Prior research has suggested that ESWL treatment may induce new-onset diabetes [21]. It has been found that after a mean follow-up of 13.7 years in 2 643 cases, the risk of new-onset diabetes in patients with urinary calculi treated with ESWL was significantly increased, and the impact did not alter with the change of the calculus site treated with ESWL [22, 23]. Patients with distal ureteral stones far away from the pancreas suffer an increased risk of new-onset diabetes after ESWL. Another clinical study with a 15-year follow-up showed that only patients with an intensity > 15 KV during ESWL treatment resulted in increased fasting blood glucose after treatment and an increased chance of new-onset diabetes [24, 25]. However, the present study failed to analyze the impact of diabetes in the treatment efficacy. Hence, further studies with more clinical data are warranted to clarify the mechanism of diabetes in urinary calculi.

The article "The Clinical Efficacy and Safety of Extracorporeal Shock Wave Lithotripsy in the Treatment of Patients with Urinary Calculi" was retracted in 2023. Reasons: unreliable results or conclusions; lack of ethics approval or compliance; concerns about the data; concerns about the peer review.

In clinical practice, laser lithotripsy, pneumatic ballistic lithotripsy, and shock wave lithotripsy are commonly used. Shock wave lithotripsy is less invasive, has a lower risk of postoperative complications, and allows accurate determination of stone location by X-ray and ultrasound before shock wave lithotripsy to improve the efficiency and accuracy of lithotripsy. The use of pulsed energy to break up stones into small fragments that can be easily removed causes no surgical trauma and avoids the limitations of other common procedures, such as the limited operation in different parts of the bladder and ureter during pneumatic bomb lithotripsy, and the problem of incomplete removal of stones due to the limited energy of the pulses, especially when multiple stones are present.

This study is different from traditional lithotripsy. According to the aesthetic appeal of patients, we chose extracorporeal lithotripsy. It provides more concern for the further use of minimally invasive treatment and also lays a certain experimental foundation for in vivo research. This study explored the mechanism of urinary calculi and the etiology and pathogenesis of traditional Chinese medicine and also provided certain opinions for the treatment and diagnosis of urinary calculi. The study had the following shortcomings: (1) The sample size of this study was small, and the significant differences in postoperative efficacy between the two groups could not be evaluated more comprehensively and objectively. (2) The study used more subjective efficacy assessment criteria, so it was difficult to describe the scale objectively and accurately because of the differences in subjective perceptions between individuals, their different levels of education, and their understanding of the questions on the scale. (3) The follow-up after surgery was relatively short in this study. (4) No animal experiment was conducted. Although this study is only a routine clinical trial, it also provides a certain direction for future animal experiments, and it is expected that animal experiments will be conducted in the future to provide new ideas for clinical treatment.

To sum up, ESWL is effective in treating patients with urinary calculi with a simple, safe, and quick operation and a low incidence of adverse events. ESWL shortens the hospital stay, reduces intraoperative bleeding, accelerates the patient's recovery, and improves the patient's renal function.

The article "The Clinical Efficacy and Safety of Extracorporeal Shock Wave Lithotripsy in the Treatment of Patients with Urinary Calculi" was retracted in 2023. Reasons: unreliable results or conclusions; lack of ethics approval or compliance; concerns about the data; concerns about the peer review.

## Figures and Tables

**Table 1:** Comparison of baseline data ($\bar{x}\pm s$).

Groups	*n*	Gender	Age (year)	Stone location				Stone diameter (cm)
				Kidney stone	Kidney stone with ureteral stone	Ureteral stone	Bladder stone	
Observation group	45	24/21	28-69 (41.69 ± 8.17)	15	13	10	7	0.62-2.88
Control group	45	23/22	24-71 (42.08 ± 7.59)	14	12	11	8	0.64-2.81
*t*	—	—	0.235	—	—	—	—	—
*P* value	—	—	0.815	—	—	—	—	—

**Table 2:** Comparison of surgical index levels between the two groups($\bar{x}\pm s$).

Groups	*n*	Operation time (min)	Early activity time (d)	Hospital stay (d)
Control group	45	36.23 ± 2.18	38.62 ± 5.37	14.12 ± 2.68
Observation group	45	30.24 ± 2.18	30.04 ± 7.07	9.17 ± 1.21
*t*	—	9.917	6.824	11.671
*P*	—	<0.001	<0.001	<0.001

**Table 3:** Comparison of VAS scores between the two groups of patients (%).

Groups	n	Mild pain	Moderate pain	Severe pain
Control group	45	28 (62.22)	12 (26.67)	5 (11.11)
Observation group	45	40 (88.89)	5 (11.11)	0 (0.00)
*x* ^2^	—	4.204	5.123	5.248
*P*	—	0.002	0.001	0.001

**Table 4:** Comparison of the number of urine red blood cells between the two groups ($\bar{x}\pm s$).

Groups	n	Urine red blood cells (×10°/L)
Control group	45	40.78 ± 8.78
Observation group	45	41.75 ± 9.08
*t*	—	0.587
*P*	—	0.554

**Table 5:** Comparison of stone excretion time between two groups ($\bar{x}\pm s$).

Groups	n	Stone expulsion time (d)	
		Before	After
Control group	45	12.87 ± 5.19	11.98 ± 6.87
Observation group	45	5.61 ± 1.37	8.54 ± 4.17
*t*	—	8.261	2.679
*P*	—	<0.001	0.008

**Table 6:** Comparison of stone removal between the two groups (%).

Groups	*n*	Successful one-time lithotripsy	Stone clearance rate
Control group	45	32(71.11)	40(88.89)
Observation group	45	43(95.56)	44(97.78)
*x* ^2^	—	10.008	7.458
*P*	—	0.002	0.005

**Table 7:** Comparison of clinical efficacy (%).

Groups	*n*	Markedly effective	Effective	Ineffective	Total efficacy
Observation group	45	21 (46.67)	23 (51.12)	1 (2.22)	44 (97.78)
Control group	45	15 (33.34)	22 (48.89)	8 (17.78)	37 (82.22)
*t*	—	6.049			
*P* value	—	0.014			

**Table 8:** Comparison of incidence of complications (%).

Groups	*n*	Hematuria	Renal colic	Nausea and vomiting	Urinary tract infection	Other	Total efficacy
Observation group	45	2 (4.45)	1 (2.23)	1 (2.23)	0 (0.00)	1 (2.23)	5(11.12)
Control group	45	6 (13.34)	3 (6.67)	2 (4.45)	2 (4.45)	1 (2.23)	14(31.12)
*t*	—	5.404					
*P* value	—	0.020					

## Data Availability

All data generated or analyzed during this study are included in this published article.
